The article "Research on Brand Illustration Innovative Design Modeling Based on Industry 4.0" was published in 2022. Journal: Comput Intell Neurosci.

# Research on Brand Illustration Innovative Design Modeling Based on Industry 4.0

**DOI:** 10.1155/2022/7475362

**Published:** 2022-04-11

**Authors:** Yueyan Liu, Zou Ping

**Affiliations:** School of Academy of Arts, Qingdao Huanghai College, Qingdao, Shandong 266555, China

## Abstract

With China's attention to the requirements of brand illustration innovative design, under the background of Industry 4.0, the advantages of applying 3D modeling method in the field of traditional illustration design are becoming more and more prominent. Based on this, this paper studies the modeling method of brand illustration innovative design based on Industry 4.0 and constructs a 3D analysis model of illustration design based on cattle cooperative hybrid algorithm. This paper innovates the innovative design method of brand illustration under the background of Industry 4.0 from the three aspects of illustration structure, illustration style, and illustration creation method, uses the cattle cooperative hybrid algorithm to quantify its innovation, and realizes the intelligent evaluation of its innovation and the quantitative representation of modeling method based on the illustration database. The experimental results show that the illustration innovative design analysis model based on cattle collaborative hybrid algorithm can effectively combine the industrial 4.0 background, realize the modeling innovation at the three-dimensional level, and significantly improve its innovative design efficiency and modeling success rate.

## 1. Introduction

Industry 4.0 is a division based on different stages of industrial development. According to the consensus, Industry 1.0 is the era of steam engine, Industry 2.0 is the era of electrification, Industry 3.0 is the era of information, and Industry 4.0 is the era of using information technology to promote industrial change, that is, the era of intelligence. In order to improve the core competitiveness of Germany's industrial revolution, the new concept of occupation machine appeared in Germany's Industrial Expo in 2013. In recent years, most illustration design masters have made many achievements in modeling the innovative design of brand illustration. Among them, the illustration design of traditional cultural style is the main, supplemented by the illustration design style of local and national characteristics [1]. Under the background of industry 4.0, new designers gradually began to combine illustration innovative design with industrial elements, such as illustration and advanced manufacturing technology, intelligent manufacturing technology, robot technology, micro nano sensing technology, and other elements, so as to realize the innovative expression of their illustration [2]. On the other hand, with the emergence of a variety of modern 3D modeling methods, different types of brand illustration innovative design methods have gradually developed in a blowout way. The emergence of modern illustration design styles such as online illustration design scheme, multidimensional collaborative design, and two-dimensional and three-dimensional collaborative design provides a new direction for promoting “brand illustration innovative design” on a large scale [3]. Therefore, how to create more and better brand illustration works under the background of industry 4.0 has become an important feature of illustration design in China [4]. At present, although the existing illustration graphic design modeling method group provides a large number of reference design schemes, in terms of practical application, it is difficult to create more and more aesthetic illustration works in combination with the existing business characteristics of the actual brand company [5]. Under this background, combined with the background of Industry 4.0, this paper proposes a modeling method of brand illustration innovative design based on cattle collaborative hybrid algorithm and studies the application of different types of 3D modeling and data analysis methods in the field of intelligent illustration 3D design.

This paper studies the modeling method of brand illustration innovative design based on Industry 4.0 and constructs an intelligent illustration design modeling strategy analysis model based on cattle cooperative hybrid algorithm. Compared with the traditional illustration design method with cultural elements as the main creative style, the innovation of this paper is to apply the cattle cooperative hybrid algorithm to the innovative design of brand illustration. On this basis, make full use of different types of 3D modeling data and collaborative multidimensional data analysis methods. Taking industry 4.0 as the background, combined with brand characteristics, realize the optimal and innovative design of illustrations, and use a variety of 3D modeling methods to represent different types of illustration works. Combined with the current illustration innovation analysis system, intelligent design and performance of different types of brand illustration works are carried out.

This paper studies the application of industrial 4.0 background in brand illustration innovation design modeling, which is mainly divided into four chapters.  Chapter 1 briefly describes the background and necessity of this study.  Chapter 2 discusses the brand illustration design method and existing research results on the application of cattle cooperative hybrid algorithm (domestic and foreign) analysis and summary.  Chapter 3 constructs the analysis model of brand illustration innovative design based on cattle collaborative hybrid algorithm and uses the Laplace factor analysis method to create a 3D structure design method based on collaborative innovation and multidimensional analysis.  Chapter 4 evaluates the optimization analysis model of brand illustration innovative design and the innovation of illustration constructed in this paper. Test the price index, analyze the test data, and draw a conclusion.

## 2. Related Work

At present, there are many problems in promoting the innovation of modeling methods in the field of intelligent illustration 3D design, especially in the brand elements of illustration design scheme, intelligent digital combination method, and collaborative design [6]. Chang and other scholars found that the current process of brand illustration design mainly takes the cultural value of the brand as the core and rarely reflects the industrial 4.0 background as the characteristic elements. Therefore, they proposed a free design method of illustration design based on the brand value communication method [7]. Hummel and other scholars proposed that attention should be paid to the development of three-dimensional illustration design methods. Through the use of 3D animation table technique based on modern style, it reflects the more affinity and appeal in the process of illustration design. By combining virtual and real works, it reflects the value circle communication effect reflected by the brand through illustration [8]. According to the collaborative innovative design theory in illustration design, Qarariyah and other scholars put forward a new brand illustration innovative design system and intelligent integrated design scheme, analyzed the relationship between the traditional illustration design field and the integrated scheme of intelligent modern picture design, and realized its innovative and prominent design in the main features [9]. Aiming at the problem of slow modeling speed in illustration design, Ekman and Feng proposed an efficient illustration modeling method combined with intelligent collaborative hybrid algorithm based on illustration design theory. Through the analysis of illustration design effect, aesthetic requirements, and brand communication in different illustration design field schemes, multidimensional design is carried out according to its internal relevance. It realizes the efficient design of illustration at different levels [10]. Wang and other scholars put forward an illustration design module analysis method based on cloud comprehensive and unified distribution by analyzing the advertising illustration contents of multiple brands, combined with the actual illustration design methods, and aiming at the design commonalities of their internal correlation schemes. This method can effectively solve the low efficiency of illustration design, but it has limited-application scope and low data utilization [11]. Xu and other scholars combined with the illustration design culture and experience of local brands and used the deformed illustration design method to comprehensively analyze the traditional intelligent illustration design method. The results show that the illustration design field system has a good overall coordination effect and can be applied to different brand illustration designs and unconventional brand illustration innovative designs. It can effectively solve the problem of poor universality of illustration design methods [12]. Based on the traditional illustration design theory and illustration aesthetic structure design method, Li and other scholars proposed a panoramic brand illustration innovative design strategy. The results show that the strategy based on intelligent distribution of data flow can effectively reduce its comprehensive errors in the illustration design system and improve the overall illustration design effect. Later, it is optimized by combining Fourier function algorithm. The results show that the optimized method effectively reduces the differentiation problem in the process of illustration design [13]. In order to solve the problems of low efficiency of multi-illustration design cooperation and slow speed of multivariate analysis in the brand illustration innovation design system, Zhao and other scholars proposed an automatic design method of illustration design scheme based on genetic algorithm and particle swarm optimization algorithm. Experiments show that the automatic design method can effectively improve the innovative effect in the process of intelligent illustration design [14]. Aiming at the problem of low efficiency in traditional brand design methods, Deng and other scholars proposed a 3D modeling illustration design method combined with massive data information. This method can realize the innovative evaluation basis of brand illustration innovative design system by simulating the three-dimensional structure diagram in illustration design, but it has the problem of low efficiency [15].

To sum up, it can be seen that the current research on brand illustration innovative design still focuses on the traditional illustration style design and the method based on low-dimensional data analysis strategy, mainly on the brand elements, intelligent digital combination method, and collaborative design of illustration design scheme, and rarely on the effective combination of intelligent algorithm and industrial 4.0 background [16–18]. On the other hand, in the modeling and optimization of illustration design style, most illustration design modeling and analysis models need to summarize the modeling data in different ranges first and then conduct unified analysis and processing, which leads to the overall illustration design efficiency becoming very low. And there is no research on optimization design and construction of relevant models for illustration design modeling [19–22]. Therefore, the research on the modeling method of brand illustration innovative design based on industry 4.0 has important practical significance.

## 3. Methodology

### 3.1. Application of Cattle Cooperative Hybrid Algorithm in Brand Illustration Innovative Design Analysis Model

In this study, in order to better quantify the data level of the intelligent illustration design process, a cattle cooperative hybrid algorithm based on color recognition strategy is adopted [23]. When studying the laws of different types of multidimensional information data, cattle collaborative mixing algorithm is a more commonly used one. Cattle collaborative mixing, also known as multilinear collaborative regression analysis, is a dynamic research model for comprehensive analysis based on the correlation between data and data, which is often used in big data analysis, cloud model verification, and so on [24]. In essence, collaborative hybrid algorithm belongs to two classification problems. Generally speaking, it is to carry out different degrees of classification process according to different types of problems, take the minimum error as the solution standard, and finally realize the optimal solution of the results [25]. Collaborative hybrid operation is also a basic method of self-learning and updating at the data level. In the process of data updating and analysis, through the accumulation of the characteristics of different types of data, it can realize the high relevance and coupling verification so as to solve the unknown complex multidimensional operation problem.

In this study, in order to build the brand illustration innovation design modeling and analysis model, the cattle cooperative hybrid algorithm is the core key point for the data information required for processing, and its corresponding data processing type is also obtained by multidimensional analysis and corresponding matrix operation. The data analysis and three-dimensional simulation operation process of its intelligent illustration innovative design is shown in Figure 1.

### 3.2. Establishment Process of Performance Analysis Model of Intelligent Illustration 3D Design Based on Cattle Cooperative Hybrid Algorithm

This intelligent illustration 3D design model based on cattle collaborative innovation algorithm combines the industrial 4.0 background and brand influence analysis mechanism to simplify the processing of complex data in intelligent illustration 3D information. Therefore, the intelligent 3D design performance analysis model needs to analyze many factors of illustration innovation so as to judge whether there are closely related factors in a variety of data. Therefore, this method can not only use the three-dimensional data required in the process of illustration design as the reference standard, but also use these comprehensive average indicators with closely related factors for data analysis or represent the modeling and analysis factors existing in intelligent illustration design through one of them. In addition, the information carried by these multidata (three-dimensional images) to be processed cannot be seriously distorted. The data analysis process of the intelligent three-dimensional description model of brand illustration is shown in Figure 2.

In the process of brand design of illustration, there is a data object to be processed (illustration innovative design modeling feature information). This process is called modeling the illustration model. In three-dimensional space, the position sequence expression in the illustration innovative design model is

(1) $$\begin{array}{c} Z_{2}=\frac{\left(z_{2}\left(1\right),z_{2}\left(2\right),\ldots ,z_{2}\left(n\right)\right)}{2n^{2}+3n-1},\\ Z_{1}=\frac{\left(z_{1}\left(1\right),z_{1}\left(2\right),\ldots ,z_{1}\left(n\right)\right)}{n^{2}+n-1},\\ Y_{2}=\frac{\left(y_{2}\left(1\right),y_{2}\left(2\right),\ldots ,y_{2}\left(n\right)\right)}{2n^{2}+3n-1},\\ Y_{1}=\frac{\left(y_{1}\left(1\right),y_{1}\left(2\right),\ldots ,y_{1}\left(n\right)\right)}{n^{2}+n-1},\\ X_{2}=\frac{\left(x_{2}\left(1\right),x_{2}\left(2\right),\ldots ,x_{2}\left(n\right)\right)}{2n^{2}+3n-1},\\ X_{1}=\frac{\left(x_{1}\left(1\right),x_{1}\left(2\right),\ldots ,x_{1}\left(n\right)\right)}{n^{2}+n-1}. \end{array}$$

In the above formula, *x*, *y*, *z* refer to the three-dimensional coordinate information, *X*, *Y*, *Z* in the process of brand illustration innovative design refers to the design change position of brand illustration in the three-dimensional space, and *n* refers to the stacking product of feature points of different brand illustration innovative design. In this stage, in the processing of data groups with different dimensions, the simulation results of the three-dimensional space design change position with the cattle cooperative hybrid algorithm and the three-dimensional space change position without the cattle cooperative hybrid algorithm are shown in Figures 3 and 4, respectively.

It can be seen from Figures 3 and 4 that under the cattle cooperative hybrid algorithm, with the increase of data operation speed, the difference between the data operation efficiency corresponding to the illustration design style and the internal correlation of the illustration three-dimensional spatial design position information is very obvious, because with the increase of the number of cattle cooperative operations, different types of illustration modeling impact graph indicators also show the same change law, which gradually decreases, and when the threshold is smaller, the impact indicator is smaller, because the smaller the threshold is, the weaker the impact degree is, and the better the corresponding stability is. Therefore, this means that the cattle collaborative hybrid method proposed in this study can effectively improve the modeling efficiency of illustration innovative design.

After combining the cattle cooperative mixed variable function *K*(*x*, *y*, *z*) and the reinforcement machine learning mechanism rule function *L*(*x*, *y*, *z*), the position expression of the corresponding illustration background 3D design modeling is

(2) $$\begin{array}{c} Z_{2}^{\prime }=\frac{3n+5}{5n^{2}+7n-1}\frac{\left(z_{2}\left(1\right),z_{2}\left(2\right),\ldots ,z_{2}\left(n\right)\right)}{{\left(n+1\right)}^{2}K\left(x,y,z\right)+\left(n+2\right)L\left(x,y,z\right)},\\ Z_{1}^{\prime }=\frac{n+2}{n^{2}+n-1}\frac{\left(z_{1}\left(1\right),z_{1}\left(2\right),\ldots ,z_{1}\left(n\right)\right)}{n^{2}K\left(x,y,z\right)+\left(n+1\right)L\left(x,y,z\right)},\\ Y_{2}^{\prime }=\frac{3n+5}{3n^{2}+2n-1}\frac{\left(y_{2}\left(1\right),y_{2}\left(2\right),\ldots ,y_{2}\left(n\right)\right)}{K\left(x,y,z\right)+n^{2}L\left(x,y,z\right)},\\ Y_{1}^{\prime }=\frac{n+2}{n^{2}+n-1}\frac{\left(y_{1}\left(1\right),y_{1}\left(2\right),\ldots ,y_{1}\left(n\right)\right)}{K\left(x,y,z\right)+nL\left(x,y,z\right)},\\ X_{2}^{\prime }=\frac{3n+5}{3n^{2}+2n-1}\frac{\left(x_{2}\left(1\right),x_{2}\left(2\right),\ldots ,x_{2}\left(n\right)\right)}{K\left(x,y,z\right)+2L\left(x,y,z\right)},\\ X_{1}^{\prime }=\frac{n+2}{n^{2}+n-1}\frac{\left(x_{1}\left(1\right),x_{1}\left(2\right),\ldots ,x_{1}\left(n\right)\right)}{K\left(x,y,z\right)+L\left(x,y,z\right)}. \end{array}$$

The expressions of cattle cooperative mixed variable function *K*(*x*, *y*, *z*) and reinforcement machine learning mechanism rule function *L*(*x*, *y*, *z*) are, respectively,

(3) $$\begin{array}{c} L\left(x,y,z\right)=\frac{3x^{4}-3y^{2}-7z^{3}}{5x^{2}+7y^{2}+2z^{3}}\frac{zy^{2}x^{3}+xy^{3}+x^{-1}y^{-1}z^{3}}{x^{2}+y^{2}+z^{-1}},\\ K\left(x,y,z\right)=\frac{x^{4}-y^{2}-z^{3}}{x^{2}+y^{2}+z^{3}}\frac{yx^{2}+xy^{2}+xyz^{2}}{x+y+z}. \end{array}$$

*X*, *Y*, *Z* are the motion position function of brand illustration in three-dimensional space, *n* is the total number of feature points of different brand illustration innovative design schemes, and *x*, *y*, *z* are the spatial trajectory coordinate information of illustration three-dimensional design. When the set signal is different from the coordinate signal in the innovative design of illustration, combined with the analysis of signals by the function of reinforcement machine learning algorithm, the integral expression *Q*(*t*) of the correlation comparison results between different types of data is as follows:

(4) $$\begin{array}{c} Q\left(t\right)=\frac{k_{p}\left[e\left(t\right)+1/T_{1}\int_{0}^{t}e\left(t\right)\text{d}t+T_{D}de\left(t\right)/\text{d}t\right]}{x^{2}+y^{2}+z^{3}}, \end{array}$$

where *x*, *y*, *z* are the three-dimensional coordinate information in the process of brand illustration innovative design, *e*(*t*) represents the deviation, *k*_*p*_ represents the error increase of illustration three-dimensional design, and *T* represents the conventional modeling constant.

### 3.3. Application of Brand Illustration Innovation Analysis Model in Intelligent Illustration 3D Design

Before completing the first draft of different types of brand illustration schemes, in the process of illustration design for different types of brands, after optimizing the innovative design methods of illustration, it is necessary to select different innovative countermeasures and methods of illustration design in combination with the characteristics of innovative design of brand illustration. In this process, by adopting the technical methods involved in different types of industrial 4.0 brands, taking the design brand illustration innovative design scheme and illustration design field as the core modeling goal, the process of the involved illustration design field will be comprehensively evaluated and analyzed to obtain the optimal illustration modeling design scheme. In this process, the internal relevance of different types of data will be analyzed through the 3D modeling method of the brand illustration innovation design system.

Secondly, the intelligent illustration 3D design method is to mine the collected illustration data types. For unknown cattle cooperative mixed data target (innovative design styles of different types of brand illustration), carry out fuzzy search and screening to realize data mining and feature analysis of the overall process of illustration design modeling, and transform the information of different types of intelligent illustration design schemes into data information that can be recognized by the system through a certain pattern. Data mining of different brands will produce different effects. The speed simulation results of the modeling method of innovative illustration design in the traditional illustration 3D design method and intelligent illustration 3D design method are shown in Figures 5 and 6, respectively.

Finally, after completing the above links, it is necessary to accumulate and stack the data generated by modeling under the cattle cooperative hybrid algorithm; that is, it is also necessary to estimate the error degree through the computer database information and the preset automatic innovative judgment program of illustration and then deeply mine and analyze some information in the field of illustration design so as to realize the secondary analysis and error analysis of the data after the initial linear analysis. The results of the illustration modeling simulation analysis method under different disturbing factors in this process are shown in Figure 7.

As can be seen from Figures 5–7, with the increase of illustration modeling and simulation times, its internal relevance is very obvious, especially in the aspects of modeling efficiency and illustration innovation. Moreover, under different thresholds, the change trends in modeling spatiotemporal differences are relatively similar, which are gradually increasing or decreasing, but the increase ranges are different, which shows that the cattle collaborative innovation method can well reduce the differences in illustration design methods. This is because the cattle cooperative hybrid algorithm has an inevitable correlation between data decision-making and state transition in illustration design, so its difference will be very small.

## 4. Result Analysis and Discussion

### 4.1. Experimental Results of Intelligent Illustration Modeling and Design Method Based on Cattle Collaborative Hybrid Innovation Model

After constructing the performance analysis model of brand illustration innovative design, we need to evaluate its practical application effect in intelligent illustration 3D design. When evaluating the data acquisition and analysis model of illustration innovative design based on Industry 4.0, it needs to be evaluated from many aspects. According to the needs of innovative illustration design of different brands, this study proposes several indicators to evaluate micro nano flexible sensors. This paper analyzes the application effect and quality of intelligent illustration in three-dimensional design in the process of illustration design. Therefore, it is necessary to analyze the data corresponding to multiple indicators of the three groups of experiments. The preliminary analysis results are shown in Figure 8, in which the horizontal axis is the number of multidimensional data. The vertical axis is the innovative and beautiful effect of illustration.

As can be seen from Figure 8, in the process of this experiment, in the verification process of intelligent illustration 3D modeling design experiment, in this study, the above indicators can be properly classified, linear analysis and logistic regression through the observation results of known experimental object data. By deleting some unnecessary (i.e., less influential) impact indicators in the illustration design field. With the increase of the number of cycles of the conduction mechanism in the experiment, there are also great differences in the spatiotemporal delay accuracy of the illustration design structure under the corresponding collaborative innovation hybrid strategy, and the accuracy of the spatiotemporal difference of the experimental data of the three-dimensional financial structure will be higher. This is because the brand illustration innovation design analysis model of degree learning algorithm is optimized and classified according to the individual differences between different modeling 3D structures and technological innovation. Through the use of big data analysis and intelligent fusion technology, the whole process monitoring of illustration innovation models of different brands in the illustration design process is realized, and the process is represented by data. Through the big data analysis system, the source data is transmitted to the system terminal, and then through the intelligent data depth mining technology and optimal analysis scheme based on cattle cooperative hybrid algorithm, a one-to-one analysis scheme is provided for the heterogeneity influence link of illustration innovative design modeling method. The above is the construction idea of brand illustration innovative design intelligent model.

### 4.2. Experimental Results and Analysis

Among the multiple data indicators used in this experiment to evaluate the three-dimensional design of intelligent illustration, some or several indicators do have correlation or mixed relationship. In order to analyze the experimental data more conveniently, the six comprehensive evaluation indexes involved in the experimental process and the correlation coefficient between the indexes are analyzed. Through the impact evaluation and application of the results of the experimental analysis of the known 9 different types of intelligent illustration design methods and the corresponding indicators in the illustration design, the performance optimization design and fiber flexibility effect of intelligent illustration modeling are realized. The corresponding image analysis is shown in Figure 9. The horizontal axis is the number of experiments and the vertical axis is the impact evaluation factor.

According to the result analysis in Figure 9, the correlation degree between the first index and the second index is 0.97; that is, the coupling relationship between the illustration design effect and the illustration style selected by the modeling method in the illustration design is very high because there is also a positive correlation between the design style and the 3D modeling method in the corresponding brand illustration innovation design system. There is also a positive correlation between design style and 3D modeling method. The relevant test results of six different types of evaluation indicators are passed in the corresponding brand illustration innovation design system. It can well reflect the effectiveness and timeliness of illustration design modeling and analysis model based on cattle cooperative hybrid algorithm. On the other hand, the experimental results show that the correlation degree between the second index and the third index is 0.96, which is very close to 0.9, which also shows that the aesthetics and symmetry in the field of illustration design are also very relevant, and its correlation value is more in line with the current practical experience, which also shows that there is a strong correlation between the two. It can be explained that the innovative modeling of illustration design and brand is also a strong correlation of positive synergy.

Therefore, the results of this study show that the intelligent illustration 3D design method based on big data analysis strategy and cattle collaborative hybrid algorithm can realize the efficient analysis of the internal information and external correlation degree between the data generated by different brands in the illustration design process. In addition, the relationship between brand illustration innovative design effect and external aesthetics can also be quantified and compared through the design modeling analysis model proposed in this study, and the degree of correlation is very small or even negligible, which is also in line with our life experience—under the background of Industry 4.0, the relationship between brand illustration design effect and external aesthetics is not large. This also shows the accuracy and objectivity of the results of this study in the application of brand illustration innovative design Industry 4.0 based on cattle collaborative innovation algorithm in innovative design.

## 5. Conclusion

In recent years, with the vigorous promotion of Industrial 4.0 technology, the application prospect of traditional illustration design in brand 3D modeling is becoming more and more obvious. Based on this, this paper studies the modeling method of brand illustration innovative design based on Industry 4.0 and constructs an intelligent illustration design and modeling strategy analysis model based on cattle cooperative hybrid algorithm. The collection of data and information in the process of brand illustration innovative design is realized from six aspects. The cattle cooperative hybrid algorithm is used to realize its data fusion. Combined with the quantitative evaluation method of multidimensional data, the illustration intelligent analysis model can comprehensively analyze and evaluate the data of different types of models. According to the relevant requirements in the field of illustration design and the general rules of modeling design method, the efficient modeling method in the process of brand illustration design is improved. Finally, relevant experiments are designed for verification. The experimental results show that the intelligent illustration design modeling model based on cattle cooperative hybrid algorithm has the advantages of quantifiable evaluation and good stability. It can improve the efficiency of illustration three-dimensional design and strengthen the intelligence of brand illustration innovation design system. However, this study only analyzes the impact and relevance of modeling methods in intelligent illustration design and does not take other potential influencing factors in the implementation of intelligent illustration design methods into account. Therefore, the impact of other factors on the modeling effect of brand illustration innovative design needs to be further studied.

## Figures and Tables

**Figure 1:** Data analysis and 3D simulation operation process of intelligent illustration creative design.

**Figure 2:** The data analysis process of the intelligent 3D description model of the brand illustration.

**Figure 3:** The spatial position change of the illustration design at different speeds without using the herd collaborative hybrid algorithm.

**Figure 4:** The spatial position change of the illustration design at different speeds using the herd collaborative hybrid algorithm.

**Figure 5:** Simulation results of traditional illustration 3D design methods.

**Figure 6:** Simulation results of intelligent illustration 3D design method.

**Figure 7:** The results of illustration modeling simulation analysis under different disturbance factor values.

**Figure 8:** Preliminary analysis results of experiments under the cooperative hybrid algorithm of cattle herd.

**Figure 9:** Analysis of experimental results under the synergistic hybrid algorithm of cattle.

## Data Availability

The data used to support the findings of this study are available from the corresponding author upon request.
